# Using Convolutional Neural Network with Cheat Sheet and Data Augmentation to Detect Breast Cancer in Mammograms

**DOI:** 10.1155/2020/9523404

**Published:** 2020-10-28

**Authors:** Saleem Z. Ramadan

**Affiliations:** Department of Industrial Engineering, German Jordanian University, Mushaqar, 11180 Amman-, Jordan

## Abstract

The American Cancer Society expected to diagnose 276,480 new cases of invasive breast cancer in the USA and 48,530 new cases of noninvasive breast cancer among women in 2020. Early detection of breast cancer, followed by appropriate treatment, can reduce the risk of death from this disease. DL through CNN can assist imaging specialists in classifying the mammograms accurately. Accurate classification of mammograms using CNN needs a well-trained CNN by a large number of labeled mammograms. Unfortunately, a large number of labeled mammograms are not always available. In this study, a novel procedure to aid imaging specialists in detecting normal and abnormal mammograms has been proposed. The procedure supplied the designed CNN with a cheat sheet for some classical attributes extracted from the ROI and an extra number of labeled mammograms through data augmentation. The cheat sheet aided the CNN through encoding easy-to-recognize artificial patterns in the mammogram before passing it to the CNN, and the data augmentation supported the CNN with more labeled data points. Fifteen runs of 4 different modified datasets taken from the MIAS dataset were conducted and analyzed. The results showed that the cheat sheet, along with data augmentation, enhanced CNN's accuracy by at least 12.2% and enhanced the precision of the CNN by at least 2.2. The mean accuracy, sensitivity, and specificity obtained using the proposed procedure were 92.1, 91.4, and 96.8, respectively, while the average area under the ROC curve was 94.9.

## 1. Introduction

Breast cancer is the second cancer-related cause of deaths among women worldwide [1]. It occurs when abnormal cells grow in an uncontrolled manner causing proliferation of the abnormal cells. This can cause death if the proliferation forms metastasis and spread to the surrounding tissues or other parts of the body. In this case, the tumor is called malignant [2]. Breast cancer usually starts in the ducts or the glands of the breast by forming lumps that can be detected by mammograms [3]. According to the American Cancer Society, it is expected to diagnose 276,480 new cases of invasive breast cancer in the USA and 48,530 new cases of noninvasive breast cancer among women and 2,620 invasive breast cancer cases among men in 2020. The society expects that about 42,170 women will die from breast cancer in this year. Death rates have been steady in younger women since 2007. They have continued to decrease in older women since 2013 thanks to a combination of factors such as enhancing early detection capabilities through screening, increasing awareness, and improving treatments. This reduction in rates comes at the expense of increasing the demand for breast imaging specialists. Computer-Aided Diagnosis (CAD) systems for breast cancer detection and diagnosis using mammograms can help in reducing the pressure on breast imaging specialists by assisting them in classifying mammograms into normal or abnormal mammograms. A complete review of the methods used in CAD for breast cancer detection using mammograms can be found in [4, 5]. Unfortunately, a precise classification of a mammogram needs a well-trained CAD system, and this requires a large number of labeled mammograms to be used in training, which is not always available. Data augmentation can help in this respect by generating artificial data.

Recently, many researchers worked on breast cancer detection in mammograms using deep learning and data augmentation. Deep learning showed many advantages over traditional machine learning and artificial intelligence [6–8]. It is used widely in image classification and particularly in medical imaging to detect various kinds of cancers and tumors such as skin, brain, and breast cancers [9–11]. The convolutional neural network was also used in breast cancer detection. A complete technical review on CNN in breast cancer can be found in [12].  Table 1 shows a summary of some methods used in breast cancer detection using CNN. The full version of this table can be found in Table 2 of [13].

The convolutional neural network, as a discriminative supervised deep learning network, consists of many stacked convolutional layers [6, 20]. Commonly, a discriminative CNN consists of a convolutional layer, a pooling layer, a rectified linear unit (ReLU), batch normalization, a softmax layer, and a fully connected layer. These layers are aligned on the top of each other to form a deep network that can accept 2D or 3D images as the input [21]. One of the first deep networks is AlexNet, which consists of 5 convolutional layers followed by three fully connected layers and ending with a softmax layer. Each of the first two convolutional layers is followed by normalization and Max pooling layers, and a Max pooling layer follows the last convolutional layer. AlexNet used the ReLU activation function as ReLU converge faster than other activation functions such as Sigmoid or Tanh [6]. Oxford University enhanced the AlexNet by replacing the large kernel size of the filters in AlexNet by multiple 3 by 3 kernel-size filters to enhance the receptive field because multiple nonlinear layers increase the depth of the network, which enables the network to learn more complex features at a lower cost. This architecture is known as VGG, which stands for Visual Geometry Group [22]. Unfortunately, VGG requires high computational power as it requires high storage memory, and it requires high computational time, which renders it inefficient. The architecture of VGG-16 consists of 16 layers as follows: 13 convolutional layers, 5 Max pooling layers, and 3 dense layers, which sums up to 21 layers but only 16 weight layers. GoogleNet introduced the inception model as it suggests that most of the connections in the dense architecture are correlated and hence can be eliminated [23]. It used three different convolutions sizes, 5 by 5, 3 by 3, and a bottleneck 1 by 1, to reduce the computational requirements and to enhance the receptive field and to better grasp of small details. GoogleNet reduced the total number of parameters. It introduced a global average pooling convolutional layer as its last convolutional layer to average the channel values across the 2D feature map.

Unlike GoogleNet, AlexNet, and VGG, Residual Network (ResNet) is not a sequential network architecture, but it is a network-in-network architecture. It uses microarchitectures (building blocks along with pooling, convolution, etc. layers) to build a macroarchitecture. ResNet was introduced to overcome the degradation problem caused by increasing the network depth [24]. ResNet introduced blockwise skip connections in convolutional layers to construct a residual module. ResNet reduced the vanishing gradient problem via skipping one or more convolution layers, which allowed ResNet to simplify deep networks during early training by utilizing the activations of adjacent layers and expanding and utilizing the skipped layers later in training. It was argued in [25] that the performance of ResNet outperforms the performance of VGG and GoogleNet.

The drawback of all the above networks and deep learning, in general, is their need to a large number of labeled training samples to learn the patterns in the images and hence classify the images correctly, which can be difficult and costly. Unfortunately, in medical images, the amount of available labeled training data is limited [26]. Training a deep model by limited labeled training set results in overfitting as the model tends to “memorize” the training set. To overcome this issue, many researchers used 2D patch and 3D cube techniques to come up with more labeled training samples [27, 28]. Some researchers used pretrained weights and replaced the last layers by the new targeted class [29–31]. Some other researchers used trained models with small input sizes and then transformed the weights in the fully connected layers into convolutional kernels [32]. Other researchers used data augmentation to synthetically expand the amount of data available for training through applying several transformation forms to the actual data such as flipping, rotating, jittering, and random scaling to the actual data [33–37]. Data augmentation is a compelling method against overfitting as the augmented data represents a complete set of data points, which minimizes the variation between training and validation sets on the one hand and the testing set on the other hand [38–45].

Data augmentation is not without drawbacks. In the domain of medical images, data augmentation should be limited to minor changes even though it has been applied heavily in the computer vision domain [46].

The artifacts and pectoral muscle in mammograms are seen as distraction by the CNN classifier and hence must be removed. Manual cropping is usually used to isolate the regions of interest in the mammograms before feeding them to the CNN as input images. Many researchers have automated this isolation processes. In [47], the authors used genetic algorithms (GA) to determine the region of interest (ROI) automatically using the area under the receiver operating characteristic curve (AUOC) as the fitness value. The procedure used in [47] has three parts: artifact removal, pectoral muscle removal, and the best ROI determination. The artifact portion removal procedure starts by dividing the mammograms into LMLO and RMLO (left-sided and right-sided mammograms, respectively) exploiting the location of the continuous vertical white line and the black region between the artifacts and the breast region. The pectoral muscle removal procedure exploits the difference in the density between the pectoral muscle tissues and the rest of the breast. The pectoral muscle tissues are denser than the rest of the breast, and hence, the pectoral muscle tissues have higher pixel values than the rest of the breast tissues. After the pectoral muscle and the artifacts are removed, the procedure in [47] draws an imaginary rectangle enclosing the remaining part of the mammogram and records the length of the longer side of the rectangle *R*. The imaginary rectangle encloses the central part of the breast, which plays the role of the initial region of interest (IROI). *R* along with the other three parameters (a parameter for height *H*, a parameter for width *W*, and a threshold value for the pixels CutVal) are used in GA to determine the best ROI from the IROI found earlier.  Table 3 shows the chromosome representation used in this GA. The chromosome consists of 3 genes corresponding to *H*, *W*, and CutVal parameters, respectively.

This procedure can be seen as a zooming procedure that determines the most beneficial region in the mammogram ROI. One should notice that the procedure used in [47] does not require the (*x*, *y*) location of the ROI or its radius to be provided by the imaging specialist to determine the ROI. Once the value of *R* and the values of *H*, *W*, and CutVal are found, the ROI is determined automatically for the mammogram and is available to be used in constructing easy-to-recognize artificial patterns (cheat sheet data) for the mammogram before it is passed to the CNN.

In this study, we propose a novel procedure to aid imaging specialists in detecting normal and abnormal mammograms. The procedure supplies the designed CNN with a cheat sheet containing classical attributes extracted from the ROI and increases the number of labeled mammograms through data augmentation. The cheat sheet aids the CNN through encoding easy-to-recognize artificial patterns in the mammogram before passing it to the CNN, while the data augmentation aids the CNN with a complete set of data points. The rest of the paper is organized as follows.  Section 2 presents the methodology, Section 3 describes the experimentation, Section 4 discusses the results, and Section 5 concludes.

## 2. Methodology

Figure 1 shows the flow chart for the procedure used in this paper to classify the mammograms. The procedure starts with extracting the ROI from the mammogram. The ROI is determined according to the procedure explained in [47] and briefly reviewed in Introduction. The extraction of the ROI is followed by taking an electronic biopsy from it, i.e., taking random pixels from the ROI. The results of the biopsy and the radius of the ROI are encoded in the mammogram as artificial patterns by drawing two frames of 10-pixel wide (one inside the other) around the ROI. The pixels' values for the two frames are equal to the average pixels' values of the biopsy (outer frame) and the radius of the ROI (inner frame). After encoding the attributes (biopsy and radius) in mammograms, mammograms are split into two sets: testing and training. Data augmentation is done on the training set (by rotating the mammograms 90° and 180°) followed by resizing the resulting mammograms into 100 × 100 before the mammograms are input to the CNN for classification.

Figure 2 shows the ROI for mdb025 from which the electronic biopsy can be taken. ROI was determined by the procedure mentioned in [47] and briefly explained in Introduction.

Figure 3 shows two augmented mammograms generated from Figure 2 by rotating the mammogram 90° and 180°.

The average pixels' values for the electronic biopsy taken from the ROI of mdb025 mammogram is 196.9, and the radius of the ROI is 75.  Figure 4 shows the result of adding the two frames to the ROI for the mdb025 mammogram in Figure 2 using the electronic biopsy and the radius of the ROI attributes. Encoding the two attributes in the mammogram is considered as a cheat sheet to the CNN, which will aid the CNN with more patterns and hence help it to classify the mammograms better.

Figure 5 shows the ROI for mdb003 (mdb003 is a normal mammogram). One can see that the color of the outer frame surrounding the ROI is very close to the color of the region itself as there is no large difference between the pixels' values of the ROI and the corresponding average. This can be explained by the low variation in the pixels' values in the ROI for a normal mammogram, and hence, the color of the outer frame is very close to the ROI in normal mammograms.

After drawing frames for all of the mammograms, the mammograms are resized to 100 × 100 images and are fed to the CNN.  Figure 6 shows the architecture of the sequential CNN suggested in this study.

The performance of the procedure is measured using Accuracy (AC), sensitivity (SE), specificity (SP), and the area under the receiver operating characteristic curve (AUOC). The accuracy is given as follows:

(1) $$\begin{array}{c} \text{AC}=\frac{\text{TP}+\text{TN}}{\text{TP}+\text{FP}+\text{TN}+\text{FN}}, \end{array}$$

where TP is the number of mammograms correctly diagnosed as positive, TN is the number of mammograms correctly diagnosed as negative, FP is the number of mammograms incorrectly diagnosed as positive, and FN is the number of mammograms incorrectly diagnosed as negative.

The receiver operating characteristic curve (ROC) shows SE on the *y*-axis and 1 − SP on the *x*-axis. SE is the proportion of actual positive cases that are correctly identified (true-positive percentage), and SP is the proportion of actual negative cases that are correctly identified (1 − SP is the false-positive percentage). SE and SP are given by the following equations, respectively.

(2) $$\begin{array}{c} \text{SE}=\frac{\text{TP}}{\text{TP}+\text{FN}},\\ \text{SP}=\frac{\text{TN}}{\text{FP}+\text{TN}}. \end{array}$$

## 3. Experimentation

The MIAS database consists of 322 mediolateral oblique-view mammograms from which 208 mammograms are normal, 63 mammograms are benign, and 51 mammograms are malignant. For the training sets, the label 0 was given to both the 208 normal and the 63 benign mammograms, whereas the label 1 was given to the 51 malignant mammograms.

The 322 mammograms in the MIAS were randomly divided into two groups, 222 mammograms for training and 100 mammograms for testing. 25% of the mammograms in the training set were randomly assigned for validation. Four sets of experimentations were created, and 15 runs were carried out for each set to evaluate the performance of the procedure proposed in Figure 1. The first set (original set (OS)) includes the following setup: 222 mammograms for training (25% validation) and 100 mammograms for testing. The second set (data augmented set (DA)) includes 15 runs according to the following setup: 666 mammograms for training data, from which 444 were augmented by flipping the original 222 mammograms 90° and 180°. From the 666 training mammograms, 25% of them were selected randomly for validation. Moreover, 100 mammograms were selected randomly from the original 322 mammograms before data augmentation for testing.

The third set (no augmentation with cheat sheet (CS)) includes 222 mammograms (25% validation) with no data augmentation but with a cheat sheet. 100 mammograms (with cheat sheet) were selected randomly from the original 322 mammograms for testing. Both the electronic biopsy and the ROI's radius were encoded in each of the mammograms as two frames surrounding the mammogram. The fourth set (data augmentation and cheat sheet (DA/CS)) includes 666 mammograms for training data (25% validation) with data augmentation and cheat sheet from which 444 mammograms were augmented by flipping the original 222 mammograms 90° and 180°. The value of the electronic biopsy and the radius of the ROI were encoded in each of the mammograms. 100 mammograms (with cheat sheet) were selected randomly from the original 322 mammograms for testing. Table 2 summarizes the four sets used in the experimentations.

## 4. Results and Discussion

Table 4 shows the performance measures, i.e., AC, SE, SP, and AUOC, obtained for the four sets described in Experimentation and listed in Table 2.

Table 5 shows a statistical summary of the classification performance obtained for the four sets.

Figure 7 shows the ROC curves for the 15 runs obtained for DA/CS set. The average area under the ROC curve for the testing set of DA/CS is 94.9.

Figure 8 shows the normal probability plots for the accuracy obtained for the four sets. The figure shows that the accuracies are coming from normal distributions. Also, the figure suggests that the variances in the accuracies for the sets with no cheat sheet (OS and DA) are close to each other and the variances in the accuracies for the sets with a cheat sheet (CS and DA/CS) are also close to each other but with lower values than those for OS and DA. Hence, the usage of a cheat sheet reduces the variance in the accuracy, i.e., enhances the precision of CNN.

Tests of hypotheses for the ratio between two variances were carried out to verify the claim that the usage of the cheat sheet enhances the precision of the CNN. The results are shown in Table 6.

The *P* values for the different tests verify that the usage of the cheat sheet alone enhances the precision of the CNN (H01), and combining data augmentation with the cheat sheet further enhances the precision of the CNN (H02 and H03).

Figure 9 shows qualitatively that the sets with a cheat sheet (CS and DA/CS) outperform the sets without cheat sheet (OS and DA) in their mean accuracy. Moreover, the figure shows that the mean accuracy of OS and DA is close to each other while the mean accuracy of DA/CS is better than the mean accuracy of CS.

Four sets of tests of hypotheses were conducted at a significance level of 0.05 to test these claims.  Table 7 shows the results.

The *P* values confirm the claims and show that the mean accuracy for the sets with a cheat sheet (CS and DA/CS) outperforms the mean accuracy for the sets without cheat sheet (OS and DA) (H04 and H05). The mean accuracy of OS and DA is close to each other (H07), while the mean accuracy of DA/CS is better than the mean accuracy of CS (H06). This result shows that using a cheat sheet can enhance the accuracy of the CNN while using data augmentation alone does not affect the accuracy of the CNN significantly. On the other hand, using data augmentation along with cheat sheet enhances the accuracy of the CNN considerably.

## 5. Conclusions

In this study, we proposed a novel procedure to aid the imaging specialists in detecting normal and abnormal mammograms. We investigated the usefulness of aiding the CNN with classical attributes, which were extracted from the ROI, by encoding the attributes in the mammogram as artificial patterns. Also, the effect of data augmentation on the performance of CNN was investigated. Mammograms from the MIAS dataset were used in this study to show the effectiveness of the proposed procedure. The results showed that including attributes extracted from ROI in the mammograms as artificial patterns enhanced the accuracy and the precision of the CNN. Moreover, the results showed that using data augmentation alone did not affect the accuracy of the CNN significantly while combining data augmentation with artificial patterns enhanced the accuracy and the precision of the CNN considerably.

## Figures and Tables

**Figure 1:** Flow chart for the procedure used in this study to classify mammograms.

**Figure 2:** ROI for mdb025.

**Figure 3:** Data augmentation for the ROI for mdb025.

**Figure 4:** ROI for mdb025 after adding the two frames.

**Figure 5:** ROI for mdb003 after adding the two frames.

**Figure 6:** Architecture of the suggested CNN.

**Figure 7:** The ROC curves for DA/CS.

**Figure 8:** Probability plot for the accuracy obtained for OS, DA, CS, and DA/CS.

**Figure 9:** Boxplots for the four setup.

**Table 1:** Summary of some methods used in breast cancer detection using CNN [13].

Author	Method	Database	Task	Metric/value(s)
Dhungel et al. [14]	Hybrid CNNa+level set	INbreast	Mass/classification	Accuracy (0.9) and sensitivity (0.98)
Dhungel et al. [15]	CRFc+CNN	INbreast and DDSMd	Lesion/segmentation	Dice score (0.89)
Singh et al. [16]	Conditional generative adversarial network and CNN	DDSM and Reus Hospital Spain dataset	Lesion/classification	Dice score (0.94) and Jaccard index (0.89)
Agarwal and Carson [17]	CNN (scratch based)	DDSM	Mass/calcifications	Accuracy (0.90)
Gao et al. [18]	Shallow-deep convolutional neural network CNN+ResNet	Mayo Clinic Arizona, INbreast	Lesion/classification	Accuracy (0.9) and AUC (0.92)
Hagos et al. [19]	Multi-input CNN	General Electric, Hologic, Siemens	Lesion/classification	AUC (0.93) and CPM (0.733)

**Table 2:** Summary of datasets used for the experimentations.

Acronym	Description	Size of the testing set	Size of the training set	Data augmentation for the training set	Cheat sheet
OS	Original set	100	222	No	No
DA	Data augmentation	100	666	Yes	No
CS	Cheat sheet	100	222	No	Yes
DA/CS	Data augmentation and cheat sheet	100	666	Yes	Yes

**Table 3:** Chromosome representation.

*H*	*W*	CutVal

**Table 4:** The performance measures obtained for the four sets.

sOS				DA				CS				DA/CS			
AC	SE	SP	AUOC	AC	SE	SP	AUOC	AC	SE	SP	AUOC	AC	SE	SP	AUOC
75	68	78	81	79	84	80	80	92	87	95	91	93	94	97	91
85	69	78	84	69	66	73	82	90	86	89	89	92	92	97	94
75	81	75	75	83	84	82	75	91	88	90	94	89	89	97	93
80	77	80	77	77	80	86	84	86	90	92	92	94	91	96	94
69	68	81	79	78	68	85	78	89	86	89	88	92	92	98	95
77	76	77	74	75	75	83	77	89	88	90	89	91	92	96	98
80	75	83	73	78	82	81	70	87	89	93	93	94	92	95	98
77	80	80	78	76	73	79	88	90	90	91	86	93	88	96	94
81	72	76	81	69	73	83	80	89	90	91	92	94	91	98	97
74	71	77	81	72	76	83	82	85	91	95	92	90	92	99	94
80	72	74	76	77	68	75	79	89	88	93	87	93	92	96	95
77	77	77	77	83	86	77	76	87	90	93	94	91	90	94	94
77	70	78	77	76	70	80	82	89	88	92	86	94	93	97	95
85	84	79	82	72	74	82	74	90	88	90	93	93	90	98	98
77	75	84	73	75	63	86	79	85	86	91	88	89	93	98	94

**Table 5:** Statistical summary for the classification performance.

Set		AC	SE	SP	AUOC
OS	Average	77.9	74.3	78.5	77.9
	StDev.	4.1	4.9	2.8	3.4
DA	Average	75.9	74.8	81	79.1
	StDev.	4.2	7.1	3.8	4.4
CS	Average	88.5	88.3	91.6	90.3
	StDev.	2.1	1.6	1.9	2.8
DA/CS	Average	92.1	91.4	96.8	94.9
	StDev.	1.8	1.6	1.3	2.0

**Table 6:** Test of hypothesis for the ratio between two variances.

Hypotheses	*P* value and 95% CI	Conclusion
H01: the variance in the accuracy for CS equals the variance in the accuracy for OS; *σ*_CS_^2^ = *σ*_OS_^2^. H11: the variance of accuracy for CS is less than the variance of accuracy for OS; *σ*_CS_^2^ < *σ*_OS_^2^.	0.008 [0.1 ∞)	There is statistical evidence that the variance in the accuracy for CS is less than the variance in the accuracy for OS by a factor of 0.1.
H02: the variance in the accuracy for DA equals the variance in the accuracy for DA/CS; *σ*_DA/CS_^2^ = *σ*_DA_^2^. H12: the variance in the accuracy for DA is more than the variance in the accuracy for DA/CS; *σ*_DA_^2^ > *σ*_DA/CS_^2^.	0.001 [2.3 ∞)	There is statistical evidence that the variance in the accuracy for DA is more than the variance in the accuracy for DA/CS by a factor of 2.3.
H03: the variance in the accuracy for DA/CS equals the variance in the accuracy for OS; *σ*_DA/CS_^2^ = *σ*_OS_^2^. H13: the variance in the accuracy for OS is more than the variance in the accuracy for DA/CS; *σ*_OS_^2^ > *σ*_DA/CS_^2^.	0.003 [2.2 ∞)	There is statistical evidence that the variance in the accuracy for OS is more than the variance in the accuracy for DA/CS by a factor of 2.2.

**Table 7:** Quantitative analysis for observations regarding Figure 7.

Hypotheses	*P* value and 95% CI	Conclusion
H04: the mean accuracy of CS equals the mean accuracy of OS; *μ*_CS_ = *μ*_OS_. H14: the mean accuracy of CS is larger than the mean accuracy of OS; *μ*_CS_ > *μ*_OS_.	0.00 [8.56 ∞)	There is statistical evidence that the mean accuracy of the CS set is larger than the mean accuracy of OS by at least 8.56 percent.
H05: the mean accuracy of DA/CS equals the mean accuracy of DA; *μ*_DA/CS_ = *μ*_DA_. H15: the mean accuracy of DA/CS is larger than the mean accuracy of DA; *μ*_DA/CS_ > *μ*_DA_.	0.00 [13.25 ∞)	There is statistical evidence that the mean accuracy of the DA/CS set is larger than the mean accuracy of DA by at least 13.25 percent.
H06: the mean accuracy of DA/CS equals the mean accuracy of CS; *μ*_DA/CS_ = *μ*_CS_. H16: the mean accuracy of DA/CS is larger than the mean accuracy of CS; *μ*_DA/CS_ > *μ*_CS_.	0.00 [1.45 ∞)	There is statistical evidence that the mean accuracy of the DA/CS set is larger than the mean accuracy of CS by at least 1.45 percent.
H07: the mean accuracy of DA equals the mean accuracy of OS; *μ*_DA_ = *μ*_OS_. H17: the mean accuracy of DA is larger than the mean accuracy of OS; *μ*_DA_ > *μ*_OS_.	0.9 [-4.56 ∞)	There is no statistical evidence that the mean accuracy of the DA set is larger than the mean accuracy of OS.

## Data Availability

The MIAS dataset used in this study can be downloaded from https://www.kaggle.com/kmader/mias-mammography.
